The article "Effects of Physical Exercise on Physical Fitness and Mental Health of Obese Students" was retracted in 2023. Reasons: signs of a paper mill; suspected computer-generated content; unreliable results or conclusions; concerns about the data.

# Effects of Physical Exercise on Physical Fitness and Mental Health of Obese Students

**DOI:** 10.1155/2022/2347205

**Published:** 2022-08-23

**Authors:** Junfang Wu

**Affiliations:** College of Physical Education, Guizhou University, Guizhou 550025, China

## Abstract

With the rapid development of my country's economy, the rapid improvement of national living standards, the introduction of western fast food culture, and the modern lifestyle, the detection rate of obese patients in my country has increased year by year. Obesity has gradually become an important issue of social concern, especially among students, obesity is very common, seriously affecting the physical and mental health of students, and laying a hidden danger for the development of society. As an effective method, physical exercise has an important impact on the physical and mental health of obese students and has become an important way to solve the obesity problem. On the basis of a large number of literature research, this paper adopts a variety of research methods such as questionnaire survey, expert consultation, mathematical statistics and comparative analysis, and logical analysis. The current situation of extracurricular physical exercise has been investigated in detail, and after data analysis, it is found that obesity has a great negative impact on all aspects of college freshmen. The results of the study showed that the obese college students in Suzhou had a low level of physical health. The average scores of the “National Student Physical Health Standards” for boys and girls were 58.50 and 60.49, respectively, and the failure rates were 48.24% and 43.55%, respectively. Compared with the average level of college students in the whole country, the height, weight, and vital capacity of obese students in Suzhou are higher than the national level, while the vital capacity index is far lower than the national level, and there are significant differences in physical fitness items (obese girls 800 meters), standing long jump, sit-ups are higher than the national level, and there are significant differences; obese boys 1000 meters, sitting forward flexion are lower than the national level, there is a significant difference, while the standing long jump performance is slightly higher than the national level). In terms of mental health, the detection rate of various mild mental health problems among obese college students in Suzhou is as high as 44.56%, and the detection rate of various moderate mental health problems also reaches 9.69%. Compared with the national youth norm, obese college students are prone to psychological problems such as somatization, obsessive-compulsive symptoms, anxiety, terror, psychosis, hostility, and paranoia.

## 1. Introduction

Comrade Jiang Zemin pointed out in the report of the 16th National Congress of the Communist Party of China that one of the goals of building a well-off society in an all-round way is to “remarkably improve the ideological and moral quality, scientific and cultural quality and health quality of the whole nation, and form a relatively complete national education system, science and technology and cultural innovation system., national fitness and health care systems” [1]. Health quality is an important symbol of social progress and civilization, and it contains the health meanings of people's psychology, physiology, and society [2]. Put “health quality,” “ideological and moral quality,” “scientific and cultural quality” three qualities side by side, and “national fitness and medical and health system” with “modern national education system,” “science and technology and cultural innovation system” three systems side by side, which fully shows the important position of health quality, national fitness and medical and health system in the process of building a well-off society in an all-round way [3].

A healthy body is a basic premise for young people to serve the motherland and the people, and it is the embodiment of the vigorous vitality of the Chinese nation [4]. School physical education should establish the guiding ideology of health first, strengthen physical education, enable students to master basic sports skills, and develop good habits of persevering in physical activity [5]. In recent years, the state and government departments have taken a series of measures to enhance students' physique and improve their health, but this has backfired. Students' physical health has not been significantly improved. On the contrary, students' physical fitness has a significant downward trend. The phenomenon of “high and two lows” means that the obesity rate and myopia rate of students increase, and the physiological function and physical quality of students continue to decline.

Medical experts believe that obesity is a common, obvious, and complex metabolic disorder, and it is a modern civilization disease that seriously endangers human health [6]. The occurrence has an important relationship, leading to the high incidence of various diseases and shortening human lifespan [7]. Obesity is spreading globally like an epidemic, not only in developed countries such as European countries, the United States, Australia, and other countries have high and rising obesity rates, but the situation in developing countries is even more serious [8]. For example, according to World Health Organization standards, some adult Polynesians in Samoa are obese. Therefore, obesity has become an important public health problem facing the world at present, and it is imperative to prevent and treat obesity diseases [9].

According to the “Student Physical Health Standards” report of Jiangsu Province in 2008, “the proportion of overweight and obese college students has risen from the first grade to the fourth grade” [10]. Due to the general improvement of living standards, excessive intake of calories and fat, and unreasonable food structure, coupled with the lag in the publicity and popularization of nutritional science knowledge, especially the reduction of students' extracurricular exercise time, the incidence of obesity has continued to increase.

Obesity-causing behaviors involve social, biological, psychological, and other factors. Bad living habits such as smoking, diet, and lack of physical exercise may also lead to the occurrence of obesity [11]. Correcting these risk behavioral factors can effectively reduce the incidence of obesity [12]. Therefore, through the investigation and theoretical analysis of the physical health level, mental health level, and extracurricular physical exercise behavior of obese college students in Suzhou area, this study provides the theoretical basis and reference for the study of exercise prescription for public physical education, obesity prevention, and weight loss.

## 2. Theoretical Research

### 2.1. Definition and Diagnosis of Obesity

#### 2.1.1. Research on definition of Obesity

From a nutritional point of view, obesity is a manifestation of excess nutrition. It is a state in which the body's burning fat is stored in excess because the energy supply is greater than the energy consumption [13]. From a medical point of view, obesity refers to a weight state in which the number of adipocytes increases and the fat storage in adipocytes is excessive, the body fat increases excessively, the weight exceeds the normal value and causes serious harm to health [14]. From the definition of obesity, we can see that obesity refers to the excessive storage of body fat, which manifests as an increase in the number of fat cells or an increase in cell volume, resulting in a loss of normal ratio between adipose tissue and other tissues, causing the body to consume more energy than consume energy. A state.  Figure 1 shows the proportion of overweight and obesity in different age groups [15]. As can be seen from the figure, the obese people in China are mainly middle-aged aged 45–54, followed by 55–64, while the obesity rate of students aged 18–24 is small, which is mainly related to the physical function of different age groups. Because young people love exercise, and digestion ability is strong, so not easy to cause obesity.

#### 2.1.2. Research on Obesity Diagnosis

Due to the different measurement methods and measurement indicators, the scales for evaluating obesity are also different [16]. For example, by testing the two indicators of height and weight to determine the degree of obesity and height standard weight, by measuring the waist circumference and hip circumference of the two indicators waist-to-hip ratio method, as well as the underwater weighing method, skinfold thickness measurement method, bioelectrical impedance method, and body potassium determination by precision instruments to measure body composition. In the large sample research, due to factors such as cost, equipment, and time, methods such as BMI index, standard weight for height, and waist-to-hip ratio are usually used [17].

Among them, BMI is the abbreviation of Body Mass Index, which is translated into “body mass index,” “body mass index,” “obesity index,” “body mass index,” and other names in China. BMI index = weight (Kg) 1 height (m2) is an important indicator to reflect the relationship between adult weight and height and to judge the degree of body fat and thinness. It is an indicator closely related to the total amount of body fat and is widely used internationally. Assessment of relative body fatness. In 1997, WHO defined “BMI ≥ 30 Kg/m2” as obesity for adults (referred to as the international standard). In 1999, according to the characteristics of Asians, WHO defined “BMI ≥ 25 Kg/m2” as obesity in “Redefinition of Obesity and Its Treatment in Asia-Pacific Region” (referred to as the Asia-Pacific Standard). In 2002, the China Obesity Working Group Data Aggregation and Analysis Collaborative Group proposed that the Chinese “BMI ≥ 28 Kg/m2” is obese (referred to as the Chinese standard). In using the BMI index to assess the degree of obesity, it is easy to be affected by the ethnicity, age, influenced by factors such as gender, there are different judgment thresholds [18]. Although our country has established obesity standards for adults, it has not established obesity standards for the characteristics of college students.  Figure 2 shows the indicators of obesity diagnosis.

### 2.2. Overview of Physical Health and Mental Health

#### 2.2.1. Physical Health

The concept of “physical health” is expressed differently in different countries and regions. My country's neighbor Japan calls it “physical fitness,” Britain, the United States, and other countries call it “physical fitness,” and my country calls it “physical fitness” in areas other than the mainland. My country's academic circles have a wide range of research on physical health, and the concept of physical health is also constantly developing and improving. Including clinical medicine, anthropology, physical education, and other disciplines, the concept of “physical health” has been defined. In the early 1980 s, the definition of “physical health” by the Chinese Society of Sports Science was the most influential: physical fitness and individual heredity. It is highly related to the acquisition, and based on this, it shows relatively stable performance and characteristics in terms of physiological function, morphological structure, mental health, etc.. It can be seen that the concept of “physical health” includes the performance of “psychological level.” However, admittedly, in most bodies [19].

Whether abroad or at home, in schools and large-scale social group physique tests, the conditions for conducting psychological tests and adaptability are more complicated and cumbersome. Generally, physique health tests are carried out in three aspects: physical development level, physical function level, and physical quality. In my country, the physical fitness test standards and items for student groups, the “Student Physical Health Standards” (hereinafter referred to as “standards”) is the most well-known to the public and society. Based on the importance and particularity of adolescents' physical health, many countries have formulated test standards and contents for adolescents' physical health according to their national conditions. Among them, some developed countries have relatively complete systems for physical health testing of children and adolescents (students). The test items conducted in Europe and the United States are different from those in China and Japan, but they also evaluate the physical development level, physical function level, and physical fitness of children and adolescents (Table 1).

#### 2.2.2. Mental Health

In the 1890 s, psychology was officially separated from the scope of speculative philosophy and became an independent discipline. Therefore, the definition of “mental healt” was relatively late. However, the impact of mental health on individuals has long been recognized. Mental health refers to the development of an individual's psychological state into a good state within the range that the individual does not contradict others at the level of intelligence, emotion, and body. With the continuous changes in society and the gradual deepening of human's understanding of mental health, the concept of mental health has been extended and gradually deepened accordingly. One of the most obvious manifestations is the establishment of the concept that “psychology and physiology” are inseparable. On this basis, scholars from various countries have carried out in-depth research on the relationship between physiology and psychology, and also deepened the cognition of the concept of “mental health” [20].

#### 2.2.3. The Relationship between Mental Health and Physical Health

Physical fitness is an important indicator that affects the health of an individual throughout his life. It generally includes body composition indicators and physical fitness indicators (physical fitness and exercise quality), which are also called physical fitness in some countries and regions. Many studies have proved that physical health may be related to different psychological health indicators. The research on the influence of mental health on adolescent physical health mainly includes two aspects: (1) the relationship between mental health and physical development; (2) the relationship between mental health and adolescent physical development. Physical development refers to the development of the external form of the body, which is an important content reflecting the growth and development of children and adolescents and can also objectively reflect the nutritional status of individuals. Physical development is closely related to socioeconomic environment and geographical environment.  Figure 3 shows the main problems of college students' mental health. It can be seen from the figure that the main source of college students' mental health is the academic pressure, followed by interpersonal relationship and career planning. Because the main task of students is learning, the pressure caused by the learning environment and learning has an important impact on students' mental health.

## 3. The Influence of Obesity on Students' Physical Health and Mental Health and the Current Situation Investigation

### 3.1. The Effect of Physical Exercise on the Physical Health of Obese Students

Lack of physical exercise is one of the reasons for students' obesity, and to solve the obesity problem, it is necessary to participate in physical exercise. In today's society, people pay more and more attention to health, and their enthusiasm for participating in physical exercise is also rising. Physical exercise has increasingly become a social fashion. The popularity of physical exercise is due to people's deepening understanding of the important role of physical exercise in promoting physical health. For obese students, the impact of physical exercise on physical health is also very important.

#### 3.1.1. Physical Exercise Is Conducive to the Normal Development of Students

The problem of obesity means that students are not developing normally. Physical exercise can promote the normal development of students and make them healthier. The human body is composed of different systems, including the motor system, respiratory system, nervous system, blood circulation system, and digestive system. Physical exercise involves different forms of movement of various parts of the body and plays an important role in improving the functions of these systems of students. Physical exercise promotes the normal physical development of obese students by improving the function of various motor systems.

#### 3.1.2. Physical Exercise Is Conducive to the Enhancement of Physical Fitness of Obese Students

Physical quality includes strength, speed, endurance, agility, and flexibility. For obese students, there are deficiencies in these aspects, so the physical quality is poor. Physical exercise includes a lot of content and involves a lot of sports. Through the training of different sports, the strength, speed, endurance, sensitivity, flexibility, and other qualities of obese students will be greatly improved, and the overall physical fitness will be enhanced.

### 3.2. The Effect of Physical Exercise on the Mental Health of Obese Students

Mental health is an important part of health. For students, mental health is very important. It is not only related to the study of scientific and cultural knowledge, but also affects their normal life and growth. Physical exercise plays a huge role in the mental health of obese students.

#### 3.2.1. Physical Exercise can Regulate the Emotions of Obese Students

Obese students not only face huge psychological pressure in life and study, but also have various psychological problems caused by obesity. It is normal to have bad emotions.  Figure 4 shows students' body anxiety due to obesity. By participating in physical exercise, obese students can temporarily forget this kind of pressure and bad psychology in the process of sports, which is beneficial to relieve pressure and eliminate tension. In sports, obese students maintain positive emotions, optimistic and stable emotions, and in the long run, various psychological problems will be solved.

#### 3.2.2. Physical Exercise can Give Obese Students a Good Emotional Experience

Obese students will inevitably have a bad emotional experience in study and life, and physical exercise provides them with ways and means to vent. By participating in physical exercise and completing different sports tasks, obese students can gain a sense of achievement and psychological satisfaction. This kind of good emotional experience brought by physical exercise is helpful for obese students to actively face study and life and enhance their self-confidence.

#### 3.2.3. Physical Exercise can Cultivate the Strong Will of Obese Students

For obese students to participate in physical exercise, they need to master certain techniques. Learning some techniques is not easy and requires to overcome many difficulties. In the process of physical exercise, they will also face a variety of harsh environments and strong opponents, which are full of challenges. Obese students may need to challenge the limits of their bodies. In the process of constantly overcoming difficulties, completing sports tasks, and obtaining good sports performance, obese students will gain hardships and stand hard work, brave struggle, perseverance mental strength, so as to cultivate its strong will.

### 3.3. Current Situation Survey

In this paper, the physical health, mental health, and extracurricular physical exercise behaviors of the four ordinary colleges and universities in Suzhou area: Soochow University, Suzhou Institute of Science and Technology, Suzhou Arts and Crafts Vocational and Technical College, and Suzhou Agricultural Vocational and Technical College, for the research object.

The research methods include literature research method, expert interview method, and questionnaire survey method. According to the research needs of this paper, read books on pedagogy, physical fitness, school sports, psychology, sports sociology, sports management, sports economics, sports statistics, sports culture, and other aspects to prepare the theoretical basis for this research.

According to the needs of the research, two sets of questionnaires, “College Students' Extracurricular Physical Exercise Behavior Questionnaire” and “Symptom Self-rating Scale (SCL-90)” were designed. “College Students' Extracurricular Physical Exercise Behavior Questionnaire” is designed for the research needs of obese college students' exercise prescription. The Self-rating Symptom Scale (SCL-90) is a commonly used survey tool for measuring mental health at home and abroad.

In total, 600 questionnaires were distributed, 600 were recovered, the recovery rate was 100%, of which 588 were valid questionnaires (340 for boys and 248 for girls), and the recovery rate was 98%, thus ensuring the reliability of the first-hand information.

## 4. Analysis of Survey Results and Research on Countermeasures

### 4.1. Physical Health Status of Obese College Students in Suzhou

The comparison results of physical fitness test scores and national college students are shown in Table 2. From the statistical results in Table 2, the lung capacity of obese college students in Suzhou is much higher than the national index, but the lung capacity index is far lower than the national index, and there is a highly significant difference. For adults, the heavier the weight, the greater the lung capacity, but the lung capacity is easily affected by factors such as age, gender, height, weight, and chest circumference. Because the weight of obese students is relatively large, the lung capacity index is low.

### 4.2. Mental Health and Physical Exercise Status of Obese College Students in Suzhou

Table 3 shows the detection rate of mental health problems among obese college students in Suzhou. The statistical results from Table 3 show that: (1) 262 people have psychological factor scores ≥2, and the detection rate of various mild psychological problems is 44.56%. Among them, the detection rate of boys reached 44.71%, and the proportion of mild obsessive-compulsive symptoms, interpersonal sensitivity, hostility, and other symptom factors accounted for more than 20%; while the detection rate of girls reached 44.35%, mild obsessive-compulsive symptoms, interpersonal sensitivity, and other symptoms. Anxiety symptom factor ranked the top three. (2) There were 57 people whose psychological factor score was >3, and the detection rate of various moderate mental health problems reached 9.69%.

In the comparison of the scores of the obese college students' symptom self-rating scale with the national youth norm, see Table 4. Among the obese college students' symptom factors, only the average score of interpersonal relationship and depression is lower than the national youth norm, while the other seven factors were higher than the national youth norm, and there were highly significant differences in the symptom factors of somatization, obsessive-compulsive symptoms, anxiety, and psychosis, and significant differences in the symptoms of hostility, paranoia, and phobia. This shows that obese college students generally have different types and degrees of psychological problems. Compared with people of the same age, they are more likely to have psychological problems such as somatization, obsessive-compulsive symptoms, anxiety, terror, psychosis, hostility, and paranoia.

In order to find out the difference in the mental health status of obese male and female freshmen, we used gender as an independent variable to test the significance of the difference. From the statistical results in Table 5, the total score of boys is higher than that of girls, and there is a significant difference. Among the nine factors, boys only have lower scores on depression and anxiety than girls, while the other seven factors have higher scores than girls. There are highly significant differences in somatization and obsessive-compulsive symptoms, and in hostility and paranoid symptoms. There are significant differences.

Figure 5 shows the mental subhealth status of obese students in different regions. From the statistical results in Figure 5, the average score of obese college students in rural areas is the highest, followed by obese college students in counties, and obese college students in big cities have the lowest score. This is mainly related to the level of education and family economic conditions. When college students from rural areas are facing economic and academic pressure, the phenomenon of “hardship is hidden in psychology,” and they receive relatively little support from their families, which makes the psychological pressure difficult. To timely and effective evacuation, it is easy to form psychological barriers or diseases.

A survey was conducted on students of different ages and physiques, mainly to investigate their willingness to participate in physical exercise. The results are shown in Figure 6. It can be seen from the figure that the older the students are, the more overweight and obese students are more willing to participate in physical exercise, which also shows that the students are more and more aware of the harm of obesity to the body and the importance of physical exercise.

Figure 7 shows the abnormal mental health and sub-health results of obese college students. It can be seen from the figure that although the students have been studying and living on the university campus for a year, there are still a large number of students who feel unable or difficult to adapt to the new environment, and often have disputes due to lack of communication when dealing with interpersonal relationships. It leads to emotional depression and loneliness. This situation causes students to have psychological problems such as somatization, obsessive-compulsive symptoms, anxiety, terror, psychosis, hostility, and paranoia, thus affecting their physical and mental health. This is mainly because, under the influence of exam-oriented education for a long time, schools and parents, often under the command of the baton of the college entrance examination, attach great importance to the intellectual education of students, while ignoring the cultivation of students' healthy personality.

### 4.3. Recommendations for Physical Exercise for Obese Students

Schools should create more physical exercise conditions for young people as much as possible, and teachers should use positive evaluations to encourage young people to do physical exercise in physical education activities. At the same time, respect their individual differences and explore the sports' potential of each youth. In addition, give them more opportunities to show themselves, and use their strengths to the greatest extent possible in competitions or other sports activities, so as to enhance their sports confidence and interest in physical exercise.

Parents should provide their children with as much physical activity support as possible to enhance their self-esteem and self-efficacy. Parents often promote and educate about exercise. You can use verbal encouragement or behavior to participate in physical exercise with children, and actively create a good family atmosphere for physical exercise. At the same time, it can create more sports conditions for children, let them experience the fun brought by physical exercise, help them overcome their own negative personality qualities, and reduce the sedentary time of watching mobile phones and TV.

Individual students should make reasonable use of social resources. At the same time, strengthen self-regulation, fully accept and use social support, establish a good interpersonal relationship with others, actively cultivate awareness of exercise, and actively participate in physical exercise.

## 5. Conclusion

The immaturity of psychological development and weak physical health caused by obesity make students prone to mental subhealth problems under the multiple pressures of rapid social development, which in turn restricts the healthy development of young people's physique. This paper investigates the mental health and physical health problems caused by obesity among college students in Suzhou, as well as students' participation in physical exercise. The main conclusions are as follows: (1) The physical health level of obese college students in Suzhou is relatively low, and the physical health test of boys is average. The score was 58.50, and the failure rate reached 48.24%. The average score for girls was 60.49, and the failure rate reached 43.55%. (2) The detection rate of various mild psychological problems among obese college students in Suzhou area reached 44.56% (44.71% of boys and 44.35% of girls), and the detection rate of various moderate mental health problems reached 9.69% (including 44.71% of boys and 44.35% of girls). In total, 10.29% for boys and 8.87% for girls). (3) More than 80% of the obese college students in Suzhou have a positive attitude toward sports, and a few show dislikes. Boys are significantly more motivated to participate in physical exercise than girls.

## Figures and Tables

**Figure 1:** The proportion of overweight and obesity in different age groups.

**Figure 2:** Obesity diagnostic indicators.

**Figure 3:** The main problems of college students' mental health.

**Figure 4:** Students' body anxiety due to obesity.

**Figure 5:** Psychological subhealth status of obese students in different regions.

**Figure 6:** Physical exercise participation of students of different ages and physiques.

**Figure 7:** Abnormal mental health and subhealth outcomes of obese college students.

**Table 1:** Main test methods of physical health of American and European students.

Test indicators	Eurofit	FitnessGram	Alpha-fit
Body composition	Height, weight, body fat ratio 20 m round trip	Body, weight, BMI, body fat percentage	Height, weight, BMI, waist circumference

Cardiorespiratory endurance	Treadmill exercise test, grip strength	Progressive cardiovascular endurance running	20 m round trip

Muscle strength and endurance	Standing long jump, hanging arms, crunches	Mile run, crunch, cantilever suspension push ups Improved pull-ups torso up	Grip, standing long jump

Athletic ability	Run back and forth Slab undulation		4 × 10 m round trip

Coordination	Sitting forward bend	Single leg sitting forward bend	

Balance	Flamingo balance test	Shoulder stretch	

**Table 2:** The statistical table of comparison between the physical health test scores of obese college students in Suzhou area and the national college students.

Gender	Boy		Girl	
Project	Sample (340)	National	Sample (248)	National
Height	174.79 ± 5.80	171.02 ± 6.06	163.20 ± 4.7	159.48 ± 5.44
Weight	81.10 ± 8.84	61.24 ± 9.09	70.10 ± 5.57	51.28 ± 6.57
Lung capacity	4302.51 ± 676.08	3727.56 ± 729.26	3025.32 ± 450.87	2445.28 ±562.54
Spirometry index	53.44 ± 8.88	61.47 ± 11.76	43.35 ± 6.894	48.04 ± 10.92
Standing long jump	230.33 ± 16.99	228.84 ± 19.67	170.92 ± 14.71	168.96 ± 17.94
Sitting forward bend	11.47 ± 4.81	12.46 ± 7.23		
Sit-ups			34.12 ± 7.88	31.43 ± 9.19
1000 meters	259.69 ± 29.05	256.29 ± 32.05		
800 meters			243.81 ± 21.15	254.53 ± 30.13

**Table 3:** Detection rate of mental health problems in obese college students in Suzhou area.

	Factor score		Total	Factor score		Total
	Boy	Girl		Boy	Gril	
Overall	152	110	262	35	22	57
Somatization	50	22	72	4	2	6
Obsessive-compulsive symptoms	112	80	192	8	7	15
Interpersonal relationship	84	64	148	14	7	21
Depression	44	34	78	8	2	10
Anxiety	40	44	84	6	2	8
Hostility	78	32	110	4	13	17
Fear	34	24	58	8	0	8
Paranoid	56	34	90	12	4	16

**Table 4:** Comparison of the scores of the obese college students' symptom self-rating scale with the national youth norm and the national college student norm.

	Tested college students	National youth norm	National university student norm	T1	T2
Somatization	1.47	1.34	1.57	5.359	−4.757
Obsessive-compulsive symptoms	1.84	1.69	2.03	4.902	−7.618
Interpersonal relationship	1.72	1.76	1.92	−1.202	−7.610
Depression	1.54	1.57	1.91	−1.047	−16.598
Anxiety	1.51	1.42	1.68	3.733	−7.844
Hostility	1.57	1.50	1.73	2.342	−6.252
Fear	1.39	1.33	1.54	2.367	−6.870
Paranoid	1.58	1.52	1.84	1.977	−10.547
Psychotic	1.49	1.36	1.61	5.518	−6.020

**Table 5:** Comparative statistics of psychological symptoms characteristics of obese college students of different genders.

	Boy	Girl	T
Overall	142.68	138.10	1.976
Somatization	1.52	1.39	3.704
Obsessive-compulsive symptoms	1.89	1.78	2.638
Interpersonal relationship	1.75	1.69	1.289
Depression	1.54	1.55	-0.270
Anxiety	1.50	1.52	-0.541
Hostility	1.61	1.52	2.056
Fear	1.40	1.37	0.808
Paranoid	1.62	1.52	2.370
Psychotic	1.51	1.47	1.219

## Data Availability

The labeled data set used to support the findings of this study is available from the author upon request.
